# Critical research gaps and translational priorities for the successful prevention and treatment of breast cancer

**DOI:** 10.1186/bcr3493

**Published:** 2013-10-01

**Authors:** Suzanne A Eccles, Eric O Aboagye, Simak Ali, Annie S Anderson, Jo Armes, Fedor Berditchevski, Jeremy P Blaydes, Keith Brennan, Nicola J Brown, Helen E Bryant, Nigel J Bundred, Joy M Burchell, Anna M Campbell, Jason S Carroll, Robert B Clarke, Charlotte E Coles, Gary JR Cook, Angela Cox, Nicola J Curtin, Lodewijk V Dekker, Isabel dos Santos Silva, Stephen W Duffy, Douglas F Easton, Diana M Eccles, Dylan R Edwards, Joanne Edwards, D Gareth Evans, Deborah F Fenlon, James M Flanagan, Claire Foster, William M Gallagher, Montserrat Garcia-Closas, Julia M W Gee, Andy J Gescher, Vicky Goh, Ashley M Groves, Amanda J Harvey, Michelle Harvie, Bryan T Hennessy, Stephen Hiscox, Ingunn Holen, Sacha J Howell, Anthony Howell, Gill Hubbard, Nick Hulbert-Williams, Myra S Hunter, Bharat Jasani, Louise J Jones, Timothy J Key, Cliona C Kirwan, Anthony Kong, Ian H Kunkler, Simon P Langdon, Martin O Leach, David J Mann, John F Marshall, Lesley Ann Martin, Stewart G Martin, Jennifer E Macdougall, David W Miles, William R Miller, Joanna R Morris, Sue M Moss, Paul Mullan, Rachel Natrajan, James PB O’Connor, Rosemary O’Connor, Carlo Palmieri, Paul D P Pharoah, Emad A Rakha, Elizabeth Reed, Simon P Robinson, Erik Sahai, John M Saxton, Peter Schmid, Matthew J Smalley, Valerie Speirs, Robert Stein, John Stingl, Charles H Streuli, Andrew N J Tutt, Galina Velikova, Rosemary A Walker, Christine J Watson, Kaye J Williams, Leonie S Young, Alastair M Thompson

**Affiliations:** 1 Imperial College London, Exhibition Rd, London SW7 2AZ, UK; 2 University of Dundee, Perth Road, Dundee DD1 4HN, UK; 3 University of Southampton, University Road, Southampton SO17 1BJ, UK; 4 University of Birmingham, Edgbaston, Birmingham B15 2TT, UK; 5 University of Manchester, Oxford Road, Manchester M13 9PL, UK; 6 University of Sheffield, Western Bank, Sheffield S10 2TN, UK; 7 Kings College London, Strand, London WC2R 2LS, UK; 8 University College London, Gower Street, London WC1E 6BT, UK; 9 Cancer Research UK, Cambridge Research Institute/University of Cambridge, Trinity Lane, Cambridge CB2 1TN, UK; 10 Newcastle University, Claremont Road, Newcastle upon Tyne NE1 7RU, UK; 11 University of Nottingham, University Park, Nottingham NG7 2RD, UK; 12 London School of Hygiene and Tropical Medicine, Keppel Street, London WC1E 2HT, UK; 13 Queen Mary University of London, Mile End Road, London E1 4NS, UK; 14 University of Glasgow, University Avenue, Glasgow G12 8QQ, UK; 15 University of East Anglia, Earlham Road, Norwich NR4 7TJ, UK; 16 University College Dublin, Belfield, Dublin 4, Ireland; 17 The Institute of Cancer Research, 15 Cotswold Road, London SM2 5MG, UK; 18 University of Cardiff, Park Place, Cardiff CF10 3AT, UK; 19 University of Leeds, Woodhouse Lane, Leeds LS2 9JT, UK; 20 Royal College of Surgeons Ireland, 123, St Stephen’s Green, Dublin 2, Ireland; 21 University of Stirling, Stirling FK9 4LA, UK; 22 University of Chester, Parkgate Road, Chester, CH1 4BJ, UK; 23 University of Oxford, Wellington Square, Oxford OX1 2JD, UK; 24 University of Edinburgh, South Bridge, Edinburgh EH8 9YL, UK; 25 National Cancer Research Institute, 407 St John Street, London EC1V 4AD, UK; 26 Queen’s University Belfast, University Road, Belfast BT7 1NN, UK; 27 University College Cork, College Road, Cork, Ireland; 28 University of Leicester, University Road, Leicester LE1 4RH, UK; 29 Princess Alice Hospice, West End Lane, Esher KT10 8NA, UK; 30 Brighton and Sussex Medical School, University of Sussex, Brighton, East Sussex BN1 9PX, UK; 31 The University of Liverpool, Brownlow Hill, Liverpool L69 7ZX, UK; 32 London Research Institute, 44 Lincoln’s Inn Fields, London WC2A 3LY, UK; 33 Brunel University, Kingston Lane, Uxbridge UB8 3PH, UK; 34 Cambridge University Hospitals NHS Foundation Trust, Hills Road, Cambridge CB2 0QQ, UK

## Abstract

**Introduction:**

Breast cancer remains a significant scientific, clinical and societal challenge. This gap analysis has reviewed and critically assessed enduring issues and new challenges emerging from recent research, and proposes strategies for translating solutions into practice.

**Methods:**

More than 100 internationally recognised specialist breast cancer scientists, clinicians and healthcare professionals collaborated to address nine thematic areas: genetics, epigenetics and epidemiology; molecular pathology and cell biology; hormonal influences and endocrine therapy; imaging, detection and screening; current/novel therapies and biomarkers; drug resistance; metastasis, angiogenesis, circulating tumour cells, cancer ‘stem’ cells; risk and prevention; living with and managing breast cancer and its treatment. The groups developed summary papers through an iterative process which, following further appraisal from experts and patients, were melded into this summary account.

**Results:**

The 10 major gaps identified were: (1) understanding the functions and contextual interactions of genetic and epigenetic changes in normal breast development and during malignant transformation; (2) how to implement sustainable lifestyle changes (diet, exercise and weight) and chemopreventive strategies; (3) the need for tailored screening approaches including clinically actionable tests; (4) enhancing knowledge of molecular drivers behind breast cancer subtypes, progression and metastasis; (5) understanding the molecular mechanisms of tumour heterogeneity, dormancy, *de novo* or acquired resistance and how to target key nodes in these dynamic processes; (6) developing validated markers for chemosensitivity and radiosensitivity; (7) understanding the optimal duration, sequencing and rational combinations of treatment for improved personalised therapy; (8) validating multimodality imaging biomarkers for minimally invasive diagnosis and monitoring of responses in primary and metastatic disease; (9) developing interventions and support to improve the survivorship experience; (10) a continuing need for clinical material for translational research derived from normal breast, blood, primary, relapsed, metastatic and drug-resistant cancers with expert bioinformatics support to maximise its utility. The proposed infrastructural enablers include enhanced resources to support clinically relevant *in vitro* and *in vivo* tumour models; improved access to appropriate, fully annotated clinical samples; extended biomarker discovery, validation and standardisation; and facilitated cross-discipline working.

**Conclusions:**

With resources to conduct further high-quality targeted research focusing on the gaps identified, increased knowledge translating into improved clinical care should be achievable within five years.

## Introduction

Globally, breast cancer is the most frequently diagnosed cancer in women, with an estimated 1.38 million new cases per year. Fifty thousand cases in women and 400 in men are recorded each year in the UK alone. There are 458,000 deaths per year from breast cancer worldwide making it the most common cause of female cancer death in both the developed and developing world [1].

In the UK, the age-standardised incidence of breast cancer in women has increased by 6% over the last decade, between 1999 to 2001 and 2008 to 2010 [2]. It is estimated that around 550,000-570,000 people are living with or after a diagnosis of breast cancer in the UK [3] and, based on current projections, this figure is expected to triple by 2040 due to an ageing population and continued improvements in survival [4]. Recent research indicates that the annual cost of breast cancer to the UK economy is £1.5bn, with just over a third of that cost (£0.6bn) from healthcare alone [5]. Yet the annual spend on breast cancer research by partners of the National Cancer Research Institute has reduced in recent years despite the level of cancer research spend being generally maintained [6].

In 2006, the charity Breast Cancer Campaign facilitated a meeting of leading breast cancer experts in the United Kingdom to explore which gaps in research, if filled, would make the most impact on patient benefit. The subsequent paper [7] has helped shape the direction of breast cancer research since that time. One overarching need identified was the ‘lack of access to appropriate and annotated clinical material’, which directly led to the formation of the UK’s first multi-centre, breast-specific tissue bank [8].

This new gap analysis represents an expanded, evidence-based follow-on developed collaboratively by clinicians, scientists and healthcare professionals. The aim is to ensure that the roadmap for breast cancer research remains a relevant, consensual and authoritative resource to signpost future needs. It builds upon the previous gap analysis by briefly reviewing the current status of key areas, critically assessing remaining issues and new challenges emerging from recent research findings and proposes strategies to aid their translation into practice. Whilst a survey of progress during the last five years is not the intention of this article, the preparatory detailed discussions and data analysis could provide the basis for such a retrospective review.

## Methods

During 2012, Breast Cancer Campaign facilitated a series of workshops, each covering a specialty area of breast cancer (Figure 1). These working groups covered genetics, epigenetics and epidemiology; molecular pathology and cell biology; hormonal influences and endocrine therapy; imaging, detection and screening; current and novel therapies and associated biomarkers; drug resistance; invasion, metastasis, angiogenesis, circulating tumour cells, cancer ‘stem’ cells; breast cancer risk and prevention; living with and managing breast cancer and its treatment. Working group leaders and their multidisciplinary teams (comprising a representative cross-section of breast cancer clinicians, scientists, and healthcare professionals) participated in iterative cycles of presentation and discussion, offering a subjective consideration of the recent relevant peer-reviewed literature. Summary reports were prepared by each group, collated, condensed and edited into a draft, which was critically appraised by an external Executive Advisory Board of international experts. This position paper highlights the key gaps in breast cancer research that were identified, together with detailed recommendations for action.

**Figure 1:** **Gap analysis methodology.** The flow chart illustrates the concept, processes and procedures devised to generate the gap analysis review.

## Results

### Genetics, epigenetics and epidemiology

#### Current status

##### Genetic predisposition

Our knowledge of the heritability of breast cancer has increased significantly since 2007. Known breast cancer genes (BRCA1, BRCA2, CHEK2, ATM, PALB2, BRIP1, TP53, PTEN, CDH1 and STK11) make up 25 to 30% of the heritability [9]. Genome-wide association studies (GWAS) and the recent international collaborative analyses have confirmed 77 common polymorphisms individually associated with breast cancer risk, which add a further 14% [9-11]. Evidence from an Illumina collaborative oncological gene-environment study (iCOGS) experiment suggests that further single nucleotide polymorphisms (SNPs) may contribute at least 14% to the heritability, leaving only approximately 50% as ‘missing heritability’ (Figure 2).

**Figure 2:** **Familial cancer genetics.** The proportion of the familial component of breast cancers that can be ascribed to specific genetic defects. The difference between June 2007 and 2013 shows the impact of genome-wide association studies (GWAS) that have now identified 77 common low-risk SNPs. Courtesy of Professor Douglas Easton (University of Cambridge). Reprinted by permission from Macmillan Publishers Ltd: Nature Genetics (45,345-348), copyright 2013.

If we assume the risk estimates for polygenic markers are log additive, the cumulative risk associated with these SNPs has a median of 9% to age 80 (95% confidence intervals 5 to 15%). In the familial setting, we have learnt that common genetic SNPs can modify the risk associated with BRCA2, which may be relevant when considering risk-reducing surgery [12,13].

##### BRCA1 and BRCA2

There is improved understanding of the function of BRCA1 and BRCA2 in relation to DNA repair and therapeutic responses. For example, BRCA2 functions in RAD51 loading and BRCA1 in countering 53BP1-mediated blocking of homologous recombinational (HR)-DNA repair; hence poly (ADP-ribose) polymerase (PARP) inhibitors have been developed and trialled against BRCA-driven cancers [14]. Several additional genes associated with breast cancer risk are part of the BRCA network and there is a clear relationship with the Fanconi pathway [9]. Genes in this network point to reduced HR-DNA repair as the mechanism underlying cancer susceptibility, although the precise functions of associated signalling proteins (for example PTEN, CHK2, ATM and N-terminal BRCA1) that relate to cancer development are unknown. Gene interactions of some higher risk alleles are recognised to be sub-multiplicative, whereas low risk alleles are log-additive [15]. Some susceptibility SNPs may function at the level of chromatin remodelling/enhancer activity related to nearby gene expression.

##### Epigenetics

Epigenetic alterations are frequent and cancer-specific methylation in circulating tumour (ct)DNA in serum can be used as an early detection biomarker, or as a prognostic indicator [16,17]. The recent ENCODE study provided a wide-ranging analysis of epigenetic marks on a small fraction of the genome [18]. The first candidate gene epigenetic risk factor that could usefully be included in breast cancer risk models (once fully validated) has been identified [19]. Epigenetic factors also provide molecular measures of long-term exposure to potentially oncogenic agents. Epigenetic alterations are reversible; preclinical and recent clinical testing of epigenetic-targeted therapies such as etinostat (a DNA methylation inhibitor) and vorinostat (a histone deacetylase inhibitor) indicate that such drugs may prove effective in combination with other therapies [20,21].

##### Psychosocial considerations

Predictive genetic testing for breast cancer predisposition genes can increase distress in the short term (which reduces over time) for those identified as gene carriers, whilst non-carriers report lower levels of concern following genetic testing [22]. A number of interventions have now been developed and tested to support the genetic testing process and have been shown to reduce distress, improve the accuracy of the perceived risk of breast cancer, and increase knowledge about breast cancer and genetics [23]. Examples introduced since the last gap analysis include education using tailored information technology to prepare women for genetic counselling [24]; interventions to support women’s decisions about whether or not to have genetic testing [25] and support for gene carriers thus identified [12].

#### What are the key gaps in our knowledge and how might they be filled?

##### Moderate risk alleles

Remaining ‘moderate risk’ alleles will be found within the short term by exome sequencing and extended GWAS studies will identify additional lower risk alleles. If up to 28% of the risk from known SNPs could be explained, while the median of the risk distribution changes little, confidence limits would change dramatically, such that the women in the top 5% at risk would have >15% lifetime risk, compared with <3% lifetime risk at the lower end. A prospective analysis will be required to show that genetic risk assessment can predict risk when combined with mammographic screening. We need to determine if or how common SNPs modify the contributions of BRCA1-associated and moderate risk genes (such as CHEK2, ATM) and whether this is influenced by oestrogen levels or risk management using, for example, lifestyle or chemopreventive approaches.

Functional implications of unclassified variants in BRCA1/BRCA2, fine-mapping of risk-associated variants (from GWAS) and understanding the functional impact of the more common SNPs such as TOX3 and the role of FOXA1 remain to be determined. Similarly, deconvoluting the functional interactions between susceptibility genes and known breast cancer-associated proteins require systems biology approaches. Can we achieve a clear clinical use of the knowledge gained by GWAS, SNP and BRCA studies by validation of risk models incorporating SNPs and moderate risk alleles (in particular in the familial setting) to improve risk management? A randomised trial for population screening with mammography stratified on individual genetic risk estimates (combined with other key risk factors) is warranted.

##### BRCA1 and 2

A scheme to define categories of risk for variants in BRCA (and other) cancer genes is needed to provide specific clinical recommendations. BRCA variants of uncertain significance occur in approximately 5% of all genetic tests for BRCA1/BRCA2 mutations [26]. A range of *in silico* and functional assays is available to provide evidence for or against a genetic variant being pathogenic. A calculation combining all lines of evidence can estimate the posterior probability that a particular gene variant is predisposing to disease. The expression of breast cancer genes in normal breast tissue and pathways that may underlie cancer risk (such as DNA damage response) could be used to identify tractable markers and to direct treatment choice. Additional BRCA-deficient human tumour cell lines and animal models of breast cancer are required.

##### Epigenetics

There is a gap in our understanding of cause or consequence between epigenetic traits and gene transcription. Translational studies are needed to investigate epigenetic patterns in clinical material and from clinical trials to identify and validate prognostic markers. The extent to which epigenetic markers can be incorporated into risk models alongside genetic and lifestyle factors is not yet known. Understanding how cancer risk factors impact on the epigenome and whether this provides a mechanism for increased risk associated with those exposures is poorly understood.

##### Psychosocial considerations

Further research is needed to support informed decision making about risk management options and to assess the psychosocial implications of changing behaviour and anxiety about cancer [27]. Interventions to support discussions with those newly diagnosed with breast cancer are being developed to improve understanding of risk to individuals and their families [28]. Interventions are also required to support conversations within the family about genetic risk and its implications, given that the onus is often on the patient [29]. Research involving women at increased genetic risk for breast cancer should assess the psychosocial impact on partners and the implications for their relationships [30]. Evidence from this research needs to inform services and direct resources to support those at increased risk of breast cancer.

### Risk and prevention

#### Current status

##### Risk estimation

We know little about the exact cause(s) of the majority of breast cancers. The major challenge for prevention is to identify women at risk as precisely as possible and then to apply measures such as chemoprevention and lifestyle changes. Current models can predict probable numbers of breast cancer cases in specific risk factor strata, but have modest discriminatory accuracy at the individual level [31]. The publication of more than 70 common genetic susceptibility factors via large-scale collaborative efforts [10,32] and the realisation that mammographic density is a major risk factor is important, but the major gap in our knowledge is how to incorporate these factors into our current risk prediction models [33].

Automated methods for estimation of mammographic density require further evaluation for its potential use as a biomarker for risk stratification in screening and changes in density as a biomarker of responsiveness to preventive approaches. Studies of chest irradiation for lymphomas and carcinogens in rodent models suggest the importance of exposure to radiation during puberty [34,35].

There is a need to assess the value of several new approaches to discovering biomarkers including adductomics, transcriptomics, metabolomics [36] and epigenomics and to determine how well-established measurements (for example oestrogen levels) can be incorporated into risk models [37].

##### Chemoprevention

An overview of all trials of selective oestrogen receptor modulators (SERMs) as chemopreventive agents indicates that risk is reduced by 38% for up to 10 years from the start of five years’ treatment [38]. An issue is predicting those women who will benefit from SERM treatment. Lasofoxifene appears to be the most active SERM and its further development is desirable [39]. In postmenopausal women, the MA P3 trial indicated that exemestane reduced risk by 65% after 35 months median follow-up [40] requiring confirmation with additional aromatase inhibitor (AI) prevention studies. The value of low-dose tamoxifen and fenretinide also needs to be established [41]. Since SERMs and AIs reduce only oestrogen receptor positive (ER+ve) disease, there is a need for agents to prevent ER negative (ER-ve) disease, to distinguish between ER- and progesterone receptor (PR)-related disease [42] and to develop better animal models [43]. There is a need to confirm that oestrogen-only hormone replacement therapy (HRT) reduces risk whereas combined HRT increases risk in the Women’s Health Initiative (WHI) trials and to establish the mechanism of this dichotomy [44,45].

##### Lifestyle changes

Most studies related to breast cancer risk and lifestyles are observational. Favourable changes in lifestyle including reduction of calorie excess, increasing exercise, reducing alcohol intake and less environmental exposures to disturbance of circadian rhythm could reduce breast cancer by one third [46-49]. Communicating the potential benefits of lifestyle change, identifying teachable moments and using health services to endorse lifestyle change for prevention will require additional studies to determine why health beliefs translate poorly into action [50].

##### Weight

Marked adult weight gain in premenopausal women is associated with a doubling of risk of postmenopausal breast cancer compared with no or little weight gain [51]. Conversely, weight loss of 3kg or more is associated with a 25 to 40% reduction of cancer in older women compared with those who continue to gain weight. [52-54]. It is not clear whether to focus on all overweight women, those with gynoid or abdominal obesity or those with metabolic syndrome. Weight gain after surgery for breast cancer increases risk of relapse [55]; there is a need for further randomised trials to determine whether reducing weight in the overweight, or preventing weight gain after surgery prevents relapse. Weight management strategies seeking efficacy in the long term may be particularly difficult to sustain.

##### Diet

The effect of individual components of diet is controversial. The risk of ER-ve tumours may be reduced by high vegetable intake [56] while lowering fat intake may reduce both breast cancer risk and relapse after surgery. However, two of the three randomised trials of lower fat intake are confounded by concomitant weight loss [57,58] and the one study without weight loss showed no effect of reduction of fat intake on breast cancer relapse after surgery [59].

##### Exercise

There is evidence for breast cancer prevention with habitual exercise [60]. Observational evidence shows that a physically active lifestyle after cancer treatment prevents relapse and reduces the risk of all-cause mortality [61]. The optimal exercise regime and timing are uncertain and randomised trials are required to assess the preventive benefits. There is a need to understand the mechanism of the apparent beneficial effects of caloric restriction and exercise.

Effective and sustainable lifestyle changes (diet, exercise and weight) need to be agreed and effective routes to initiation and maintenance identified. Further work needs to be undertaken in chemoprevention strategies and adherence to effective agents.

#### What are the key gaps in our knowledge and how might they be filled?

##### Risk estimation

Prospective cohort studies are needed to develop and validate risk models, which may need to incorporate polygenic risks, mammographic density and measures of body composition. Risks may be refined by the discovery and validation of novel biomarkers such as epigenetic markers [19] and prospective validation of known markers such as serum oestrogen [62,63]. Effectiveness and cost-effectiveness, analyses to evaluate possible personalised screening and prevention programmes [64] and pilot studies to evaluate delivery options followed by large randomised trials are required. Polygenic and other biomarkers should be used to distinguish between the development of ER +ve, ER+ve/PR +ve and ER–ve cancers.

Many breast cancers arise in women without apparent risk factors; current studies suggest that polygenic risk factors and mammographic density add only a little to the Gail model [65]. Precision is required using polygenic approaches to decide whether or not to give preventive tamoxifen. Currently, about 10% of breast cancers arise in women with a 10-year risk above 5%. Taking this at-risk group and increasing the frequency of screening would be of some benefit, but more effective risk-adapted screening will depend upon a better definition of risk.

##### Screening

Further improvement and cost-effectiveness of the NHS breast cancer screening programme could include tomography, ultrasound and automated methods for the measurement of volumetric mammographic density (using software programs such as Quantra or Volpara) and automatically using these for risk stratification to adapt screening interval to risk. Experimentally, there are now opportunities for determining whether high breast density alters the response of breast epithelial cells to DNA damage or oncogene activation. This may provide prognostic value if we can define novel biomarkers to distinguish which women with high mammographic density will develop cancer [66,67].

##### Chemoprevention

Uptake of tamoxifen and raloxifene is variable and optimal methods need to be developed to explain risk, the benefit/risk ratio of treatment and to identify women who will benefit. The benefit from tamoxifen may be determined by changes in mammographic density [68] but needs confirmation. Identification of women who could develop ER-ve tumours should become possible (for example by polygenic scores). Work is required to corroborate the efficacy of lasofoxifene; the use of AIs in the preventive setting should be clarified by the International Breast Cancer Intervention Study II (IBIS II) trial, while the use of low-dose tamoxifen and retinoids also await trial results. Further studies are required to develop new preventive agents; those which might be pursued further include rexinoids, omega 3 fatty acids, sulphorophane, antiprogestins and insulin-like growth factor 1 (IGF1) inhibitors [409].

The widespread introduction of preventive agents depends upon efficient methods for identifying risk and effective counselling. Neither has been widely taken up, particularly in postmenopausal women, but the recently published NICE guidelines may signal a change for the use of tamoxifen in chemoprevention. Identification within screening programmes may be a valid approach [64]. However, since trials of chemoprevention require long duration and are costly, the development of biomarkers as indicators of effectiveness and their acceptance by regulatory agencies is attractive.

##### Lifestyle change for breast cancer prevention

A precise definition of interventions for diet and exercise and the relative importance for reduction of ER+ve or ER-ve breast cancer is unclear. The effect of caloric restriction by age and the duration of interventions remain unknown as do the underlying mechanisms of action. Identifying successful methods to translate prevention evidence into public health policy including effective behaviour change programmes and convincing clinicians to change practice in favour of prevention are required. Most evidence for lifestyle change is observational and confirmatory data from prospective randomised controlled trials (RCTs) with long-term follow-up and clinical endpoints may be needed. A breast cancer prevention trial using exercise would require a sample size of 25,000 to 35,000 and an eight to ten-year follow-up to observe a 20 to 25% decrease in risk for a moderate-to-vigorous physical activity programme. Such a large-scale study is not currently possible so the focus has been on a RCT of exercise in breast cancer patients to determine how exercise influences survival. The AMBER cohort study in 1,500 breast cancer patients measures physical activity, fitness and other indicators to determine exactly how physical activity influences survival [69].

Nevertheless, the beneficial effects demonstrated in randomised trials to prevent diabetes and cardiovascular disease need to be balanced against the enormous size and cost that would be required for such trials in breast cancer. For secondary prevention of disease recurrence after surgery, trials are due to report on caloric restriction and exercise in 2014 and 2018 [70,71].

There are teachable moments within the breast screening programmes for links to prevention through changes in lifestyle [50,64]. Reduction in alcohol consumption using community/class/cultural approaches, analogous to those for smoking, needs to be explored using social marketing approaches within a research context. It is likely that energy restriction and exercise will not be a complete answer to prevention and efforts should be made to design lifestyle prevention trials with and without energy restriction mimetic agents such as mTOR inhibitors, resveratrol, and metformin. mTOR inhibitors such as everolimus (RAD001) are effective in advanced breast cancer [72] although toxicities will prevent its use as a preventive agent; rapamycin in animal models reduces tumour incidence and increases longevity [73]. There is a need to translate these important findings into the clinic, perhaps by low dose or intermittent regimens to avoid toxicity [74]. Metformin is in clinical trial as an adjuvant for breast cancer treatment and demonstration of effectiveness in this situation could lead to assessment for prevention including in prediabetic populations [75].

### Molecular pathology

#### Current status

##### Breast cancer classification and issues of heterogeneity

During the last five years several high-profile studies have significantly advanced the molecular subclassification of breast cancer (reviewed in [76] and [77]). Intratumoral heterogeneity in both pre-malignant and invasive breast cancer is well documented. It is likely that both genetic and epigenetic instability, combined with microenvironmental and therapy-induced selective pressures lead to clonal evolution, which continues during metastatic progression. However, whether heterogeneity arises from cancer stem cell plasticity and a hierarchy of aberrant differentiation or stochastic events is a moot point (Figure 3). Genomic studies have been used to develop both prognostic biomarkers and to identify biomarkers to predict response to therapy. Nevertheless, ‘driver’ genetic changes in breast cancer will need to be filtered from the background, clinically inconsequential changes [78].

**Figure 3:** **Tumour heterogeneity. (A)** Recent molecular and genetic profiling has demonstrated significant intratumoural heterogeneity that can arise through genomic instability (leading to mutations), epigenetic events and/or microenvironmental influences. The stem cell hypothesis proposes that tumour-initiating cells are pluripotent and can thus give rise to progeny of multiple phenotypes; alternatively heterogeneity could be due to stochastic events. Temporal heterogeneity can be exacerbated by therapy (theoretically due to clonal evolution as some clones are eliminated whilst others expand). The significant molecular/genetic differences between cells in different areas within individual cancers, between primary and metastatic tumours (and potentially between cancer cells that successfully colonise different organs) have implications for the reliability of primary tumour biopsies for diagnosis, seeking biomarkers for treatment planning and responses to therapy. In addition, there is substantial inter-tumour heterogeneity. **(B)** shows images of two patients who presented with breast cancers of identical histological type and biochemical parameters. Four years later, one patient is clear of disease, while the other has evidence of multiple distant metastases, illustrative of between-patient heterogeneity in terms of response to therapy (clinical images kindly provided by Professor William Gallagher, with thanks to Dr Rut Klinger and Dr Donal Brennan (UCD Conway Institute).

Exploring the diversity and inter-tumour heterogeneity of breast cancer has led to the development of a novel classification that integrates genomic and transcriptomic information to classify 10 subtypes with distinct clinical outcomes [79]. Triple-negative breast cancer (TNBC) in particular is now recognised to demonstrate heterogeneity at the molecular, pathological and clinical levels. [80]. Such analyses, together with advanced next-generation sequencing have significant implications for improved understanding of basic tumour biology and will potentially enable the identification of new molecular targets for personalised treatment plans [81,82] Additionally, identification of non-coding RNAs is showing potential in diagnosis, prognosis and therapy [83].

##### Microenvironmental influences and tumour - host interactions

Breast development is critically reliant upon cell polarity [84], choreographed cell death pathways and interactions between epithelial cells and stroma; all processes which when deregulated are implicated in oncogenesis and tumour progression [85-87]. The tumour microenvironment, comprising a community of both malignant and non-malignant cells, significantly influences breast cancer cell behaviour [88,89]. Recently, progress has been made in understanding the bidirectional interplay between tumours and surrounding stromal cells/extracellular matrix (ECM), which can potentiate resistance to targeted therapies including endocrine therapy [90,91]. Consequently, components of the tumour microenvironment may represent targets for therapeutic intervention alongside the tumour to improve response to treatment [92].

Hypoxia reflects dynamic microenvironmental conditions in solid tumours, limits responses to radiotherapy [93] and some chemotherapeutic and anti-endocrine agents [94,95], drives genomic instability and is generally associated with progression to invasive/metastatic disease [96,97]. Tumour-stromal interactions change under hypoxic conditions to promote tumour progression via the activity of enzymes such as LOX [98], angiogenic factors and infiltrating macrophages [99,100]. A stem-like breast cancer cell subpopulation with an epithelial-mesenchymal transition (EMT) phenotype is expanded during repetitive hypoxia/reoxygenation cycles [101]. Hypoxia also contributes to cancer stem cell plasticity and niche formation [102] potentially explaining the relationship between hypoxia and chemotherapy resistance [103]. Finally, at the physiological level, host metabolic, inflammatory and immunological factors can impact on cancer development and progression, and these processes are further modified by the physical environments in which we live (Figure 4).

**Figure 4:** **Microenvironmental influences on breast cancer.** Breast cancer biology, progression and response to therapy is influenced at many levels from epigenetic effects on gene expression (for example methylation) through soluble and cell-mediated stromal interactions, intratumoural inflammatory and angiogenic components, hypoxia, host endocrinological and immunological status through to exposure to multiple agents in the environment in which we live.

#### What are the key gaps in our knowledge and how might these be filled?

##### Normal breast development and the origins of cancer

It is not known how many breast epithelial cell subpopulations function as stem cells (capable of self-renewal) or progenitor cells (which proliferate expansively) [104-106]. Clearer understanding of cell lineages, changes in transcription factor expression during breast development and definition of the nature of stem and progenitor cells is fundamental to delineating relationships between normal and malignant cells.

Current cancer stem cell (CSC) assays have limitations: dormant cells cannot be detected and cell subpopulations that give rise to clones *in vivo* may not be active in ‘mammosphere’ cultures. There is no clear consensus on markers that define functional breast CSC in mouse and human. Indeed, they may not represent a fixed subpopulation, but instead exist in specific niches in flexible equilibrium with non-CSCs, with the balance depending on interactions between them as well as external selective pressures [107-109]. Understanding this plasticity [110] and its therapeutic implications are key areas for future investigation.

##### Breast cancer subtypes: genomics and bioinformatics

Several large-scale, cross-sectional, integrated molecular studies have established comprehensive molecular portraits of invasive primary breast cancers [111-114]. The International Cancer Genome Consortium (ICGC), The Cancer Genome Atlas (TCGA) and individual studies have released sequence data; however, gaining access to and interrogating this information requires expert bioinformatic collaborations. Relating these advances in genomic knowledge to improving clinical care has yet to be achieved. Knowledge of genetic, epigenetic and host factors underpinning distinct subtypes of breast cancer (plus their associated aberrant signalling pathways) and predictive biomarkers will be essential in targeting new therapeutic agents to the right patients.

For ductal carcinoma *in situ* (DCIS), an increased understanding is required of molecular markers of prognosis, thus providing key information to avoid overtreatment. We need to know which DCIS lesions will recur if adequate surgery is performed with wide, clear margins. Biological markers of DCIS should aim at defining which lesions are likely to progress, in order to avoid radiotherapy or even surgery if the risk of invasive cancer is sufficiently remote [115]. Markers for response to radiotherapy or endocrine therapy and the need for these therapies (particularly in low-risk patients) remain unclear.

##### Tumour microenvironment and stromal influences

Paget’s venerable ‘seed and soil’ analogy - recognising that tumour-initiating cells require a permissive host environment to thrive - is beginning to be deciphered at the molecular level. [42]. The composition and biophysical characteristics of the breast matrisome [116] and how it controls different stages of gland development and in early breast cancer requires definition. It is important to identify the transcription factors that define luminal and myoepithelial cells and to understand whether additional microenvironmental factors such as the ECM and fibroblast growth factor (FGF), Notch or Wnt signalling can switch their fate. Specialised niches defined by specific cell-cell/cell-matrix interactions in the microenvironment together with soluble, ECM-bound and microvesicle-associated host factors regulate CSC activation [117]. Further research on such CSC niches, their role in dormancy and the complex relationships between CSCs and metastasis is essential [118-120].

Stromal changes predict early progression of disease [121] and in-depth knowledge of how these conditions can be manipulated for therapeutic benefit is required [122]. Advances in the field of mechanotransduction are shedding light on the mechanisms by which altered matrix density or ‘stiffness’ can influence cell behaviour, and enzymes such as lysyl oxidases (LOX) are potential targets for therapy [123].

There is a need for better biomarkers of hypoxia including gene expression profiles [124] serum proteins, circulating tumour cells (CTCs) or functional imaging that could be used non-invasively in patients to enable more rigorous testing of its prognostic/predictive value. Although hypoxia-targeted therapies have proven disappointing to date, new approaches are emerging. In common with other targeted therapies for systemic disease, methods for measuring efficacy will need to be redesigned [124-126].

Tumours have an increased dependence on aerobic glycolysis. We need to understand how hypoxia affects the tumour metabolome and thus may determine therapeutic responses [96]. The dependence of metabolically adapted breast cancer cells on altered biochemical pathways presents new therapeutic targets linked to aerobic glycolysis, acidosis and the hypoxic response [127,128]. Since these pathways also interact with classical survival and proliferation signalling pathways via PKB/mTOR, there are opportunities to develop new combinatorial therapeutic strategies.

### Breast cancer development and progression

#### Current status

##### Mammary stem cells

There is increased understanding of stem cell hierarchies and their potential roles in breast development [129-131], but debate continues on the relationship between normal stem and progenitor cells, their dysregulation in cancer and the nature of putative CSCs [132-135]. Most data suggest that breast CSCs are a defined population with basal-like or mesenchymal-like features [136-138]. There is emerging data from cell line models that the CSC state is dynamic and can be induced by the tumour microenvironment [110], and this requires further investigation in human cancers. It is not known whether there are differences in CSC phenotype between breast cancer subtypes such as luminal vs. TNBC [139,140]. An emerging consensus is that CSCs initiate metastases and tumour regrowth after therapy, but do not necessarily generate the majority cell population in primary tumours.

##### Circulating tumour cells

Blood-borne tumour cells are routinely identified in breast cancer patients but their scoring can depend upon the method used [141]. Their relationship to disseminated tumour cells (DTCs) in tissues is unclear, although a recent publication showed that the presence of CD44+CD24^-/lo^ cells (putative CSCs) in the bone marrow is an independent adverse prognostic indicator in patients with early stage breast cancer [142]. A population of CTCs from patients with primary luminal cancer (expressing EPCAM, CD44, CD47 and MET) generated multi-site metastases when injected into mice. Hence it is likely that a subset of CTCs have metastatic potential [143], which may equate to CSCs. CTCs may occur in heterogeneous emboli of multiple cell types; perhaps those containing stem-like cells and/or ‘feeder’ cells are more likely to survive and grow at distant sites.

##### Metastasis

This key hallmark of breast cancer occurs when cancer cells access lymphatic and vascular systems, enabling dissemination via lymph nodes and then via the venous and arterial vascular system to distant organs. Once the disease has spread, it becomes life-threatening and patients require systemic treatment. Metastatic relapse typically occurs many months to decades after surgery, thus we need a greater understanding of the processes that occur following tumour cell dissemination, including the phenomenon of dormancy. Recent mathematical modelling using relapse data has provided interesting insights and proposals for hypothesis testing [144]. CTCs and DTCs that generate metastases are, by definition, tumour-initiating cells; hence their study needs to relate to CSC research [145,146]. Since the last gap analysis, there has been a paradigm shift in this area with the discovery of ‘pre-metastatic niches’ (analogous to stem cell niches) in organs destined to develop metastases [147,148].

In addition, seminal research using animal models has identified tumour and host genes associated with metastatic capacity (quite distinct from tumorigenic potential), and also organotropism [149-151]. The relevance of these experimental observations to human breast cancer and the translation of these findings into clinical studies require confirmation but may provide additional predictive value [152].

Reversible EMT, regulated by many factors including transforming growth factor beta (TGFβ) signalling, Slug and Snail transcription factors and hypoxia may be linked to invasion, dissemination and drug resistance [153-156]. The role of EMT in human cancer metastasis is still controversial and the underlying molecular mechanisms are not fully understood [157]. However, mesenchymal/stromal gene signatures have been identified which relate to TNBC subtypes, bone metastasis and resistance to neoadjuvant therapies [158].

#### What are the key gaps in our knowledge and how might these be filled?

##### Circulating tumour cells and nucleic acids

It is unclear whether CTCs originate from primary tumours, micro-metastases or multiple primary and secondary sites. Indeed, CTCs from distant metastases can potentially reseed the primary tumour [159,160]. More research is needed to define the origins of these cells. Importantly, analysis of CTCs needs to be carried out as far as possible in the clinical context, where their biology can be correlated with patient outcomes. CTCs and ctDNA are particularly useful where accessible breast cancer material is not available, or to obtain serial samples during therapy, providing a window on response and relapse.

To enable further progress, systems and protocols for isolating and characterising CTCs need to be rigorously defined and standardised, with an analysis of whether all systems identify/isolate the same cells (or indeed all CTCs, since EMT may preclude identification using epithelial markers [141,161-163]). We need to know the proportion of live, quiescent and apoptotic CTCs, their characteristics and malignant potential and to understand their relationship to the primary tumour and whether different subsets of CTCs have different predictive value.

The use of ctDNA is increasing as a potentially useful further source of information on breast cancer biology and response to therapy [164-166]. miRNAs identified in the systemic circulation (free or exosome-associated) [167] may also serve as diagnostic or prognostic biomarkers and/or as therapeutic targets. Indeed, it has been suggested that exosomes themselves, with their emerging roles in bidirectional signalling, immune suppression, subversion of targeted therapy and potentiation of metastasis [168] could be removed (for example by plasmapheresis) for therapeutic benefit [169].

##### Metastatic disease

Metastasis is the major cause of treatment failure, but it is far from clear why some patients with apparently similar disease succumb and not others [170]. We need to identify key signalling pathways linked to organotropism [171] and to develop new therapies for micro-and macro-metastatic disease [172]. Given the multiple breast cancer subtypes (and associated oncogenic drivers), it will be important to try to align genotypes/epigenotypes to metastatic patterns, in order to predict likely sites of relapse. Treatment decisions are generally based on the profile of the primary cancer, but information about the evolution of the disease from CTC, DTC or (where possible) metastases at different sites is essential, since both gains and losses of potential therapeutic targets have been observed in these distinct tumour cell populations.

We need to understand how the host microenvironment at secondary sites influences tumour cell survival and to define similarities and differences between ‘permissive’ microenvironments in organs favoured by breast cancer cells such brain, bone or liver. We have learned a good deal since the last gap analysis about the ‘vicious cycle’ of bone metastasis, whereby tumour cell interactions within this unique microenvironment mutually promote metastatic outgrowth and bone remodelling via hormonal, immunological and inflammatory mediators. These findings need to be translated into new therapies targeting both tumour and host components [173] with the paradigm extended to other specialised sites such as brain [174].

### Current therapies

#### Current status

##### Clinical therapies

Current clinical therapies for breast cancer are offered on an individual patient basis via a multidisciplinary team and comprise surgery, radiotherapy and drug therapies targeting oncogenic processes. Selection of therapy is based on Level 1 evidence from large RCTs or meta-analyses of such RCTs [175-177]. Increasingly, correlative translational studies are integrated prospectively into clinical trials, aiming to define the optimal target population and provide insight into mechanisms of resistance. The individualisation of treatment, optimal duration of treatments, prediction of metastasis or drug resistance remain challenging and reflect incomplete understanding of the underlying biology of breast cancer. However, up-to-date guidelines are useful to determine the best therapy for individual patients [178].

Immunohistochemical (IHC) analyses for selecting therapeutic options generally lack reproducibility and standardization resulting in poor concordance between laboratories. The Quality Assurance programme for ER, PR and human epidermal growth factor receptor 2 (HER2) in the UK has to some extent addressed this, but for other biomarkers, including Ki67, there clearly remain problems. We need to develop standardised protocols for better quantification of biomarkers [179], especially optimised methods of sample collection/storage to ensure that unstable or transient biomarkers (such as phosphoproteins or histone marks) are retained. This is especially important for predictive markers such as HER2, together with those which report on the efficacy of HER2-directed therapies and other emerging targets.

Health inequalities remain in relation to treatment. Older people diagnosed with cancer are more likely to experience undertreatment, potentially having poorer clinical outcomes than younger women for example [180,181]. Indeed, there is a lack of data to inform decision making about treatment for the elderly patient with breast cancer in part attributable to their under-representation in trials, but clinical teams may make inadvertent ageist decisions [182,183]. In addition, breast cancer and its treatment can have a considerable impact on women and their families [184]. Psychological distress is common, although not inevitable, and is associated with poorer quality of life [185,186]. Regular distress screening is recommended as a core component of good quality cancer care [187,188] in order to provide appropriate support.

##### Surgery

Surgery remains the primary treatment for most women, with breast conservation (plus whole breast radiotherapy) providing similar outcomes to mastectomy. Following mastectomy, breast reconstruction should be considered, although uptake is incomplete. Axillary surgery has moved from clearance via node sampling techniques to sentinel node biopsy as the preferred means for assessment of axillary metastasis in early breast cancer. Neoadjuvant therapy, initially implemented to down-stage inoperable cancers, is increasingly used to assess drug efficacy in individuals and to reduce the extent of surgery required in good responders [189].

##### Radiotherapy

Radiotherapy is both clinically effective and cost-effective in the adjuvant and palliative settings. The Oxford overview of adjuvant radiotherapy trials [177] showed a halving of risk of first recurrence in all risk groups and favourable effects of local control on long-term survival. There is long-term confirmation of the value of boost irradiation to the site of excision after breast-conserving surgery in all subgroups, including women >60 years [190]. The long-term safety and efficacy of hypo-fractionated radiotherapy after breast-conserving surgery and mastectomy for operable breast cancer has recently been confirmed: (10-year results of Canadian [191] and Standardisation of Breast Radiotherapy (START) trials also suggesting generalisability to all subgroups of patients [192,193].

Trials of partial breast irradiation evaluating intraoperative radiotherapy in comparison to external beam radiotherapy [194,195] or brachytherapy [196] have short follow-up, but guidelines on partial breast irradiation [197,198] have encouraged off-study use of partial breast irradiation in advance of clinical trial results. Omission of postoperative radiotherapy after breast-conserving surgery in older, lower-risk women suggests the differential in local recurrence rates may be acceptable with a cumulative in breast recurrence of 2.5% in breast conservation surgery alone vs. 0.7% for surgery and postoperative radiotherapy (median follow-up 53 months age 55 to 75 years [199]) and at 10 years local recurrence, nine for conservation alone vs. 2% for surgery and radiotherapy in the =/>70 years, ER+ve group [200].

##### Decision making

Clinical decision-making tools to support individualised treatment can influence patients’ treatment choices and experiences [201] and communication training for oncology professionals is now widely available throughout the UK to improve the delivery of information and support to patients [202]. A recent national survey of over 40,000 patients with a broad range of cancers identified the fact that younger patients and ethnic minorities in particular reported substantially less positive experiences of involvement in decision making [203].

#### What are the key gaps in our knowledge and how might they be filled?

##### Overtreatment

A significant number of patients are overtreated to achieve the improved survival overall in early breast cancer, since we cannot define individual risks of disease recurrence or sensitivity to treatment. For survivors, the long-term side effects of treatment may be significant; individualised treatment so that patients only receive the treatment they require to achieve cure remains elusive. This is relevant to surgery, radiotherapy, chemotherapy and endocrine therapy.

With the widespread adoption of sentinel node biopsy (SNB)-limiting surgery to the axilla has substantially reduced arm morbidity [204]. A detailed understanding of underlying tumour biology is required to support decisions around surgical management, (for example axillary node clearance or not after positive sentinel nodes). No further axillary surgery even for one to two positive nodes [205] and the equivalence of axillary clearance to axillary radiotherapy for local disease recurrence (despite the differing morbidities) in the presence of a low disease burden [206] demonstrate further progress in this surgical setting. However, the optimal design of radiation treatment fields for SNB-positive patients is not known.

For postoperative radiotherapy after breast-conserving therapy, we do not have reliable ways of identifying low risk, particularly in elderly patients for whom radiotherapy might be omitted. While even low-risk patients have an approximately 50% reduction in first recurrence [177], the absolute gain for low-risk breast cancer patients (older age, small, ER+ve cancers) after breast-conserving surgery is very modest. We need reliable molecular markers of identifying such low-risk groups or individuals.

Further work is required to clarify whether the response to neoadjuvant chemotherapy can be used to guide the selection of patients for regional nodal irradiation [207] or whether patients who are clinically node positive before neoadjuvant chemotherapy and are converted to node negative after neoadjuvant chemotherapy on SNB require axillary nodal irradiation.

##### Individualisation of treatment

Understanding the optimal treatment strategies for an individual patient remains elusive. A number of genomic (for example Mammaprint, Oncotype Dx, PAM50) and immunohistochemical (for example IHC 4) tests have been developed to predict prognosis and latterly, response to chemotherapy; however, prospective trial evidence is still awaited [208]. Recently, serum metabolite profiling using a combination of nuclear magnetic resonance (NMR) spectroscopy and liquid chromatography-mass spectrometry (LC-MS) correctly identified 80% of breast cancer patients whose tumours failed to respond adequately to chemotherapy, showing promise for more personalized treatment protocols [209].

Increased understanding of the dynamic changes that occur over time is critical and will require repeated assessment of tumour profiles. Genomic tests predict response to endocrine or chemotherapy and those at highest risk of relapse [210-212], but prospective trials are required to determine whether axillary clearance or chemotherapy can be avoided in node-positive patients. Similarly, biological markers of radiosensitivity (tumour and normal tissue) require better characterisation and implementation into clinical strategies to allow personalisation of treatment and avoidance of late radiation-induced toxicity [213].

##### CNS metastatic disease

As a result of improved outcome for patients with metastatic breast cancer (MBC), central nervous system (CNS) metastatic disease is an increasing therapeutic challenge [214]. Optimal treatment strategies have yet to be defined including sequencing or combination of stereotactic and whole brain radiotherapy, systemic treatments, intrathecal treatment approaches for leptomeningeal disease and prophylactic interventions.

##### Bone metastatic disease

Bisphosphonates reduce the risk of developing breast cancer in osteoporotic and osteopenic women by approximately 30% and the risk of recurrence in early breast cancer when used at the time of diagnosis [215,216].The interaction between the internal endocrine environment and the effect of bisphosphonates is complex and poorly understood. While negative results overall were reported in the large UK AZURE trial [217] women more than five years postmenopausal benefitted, consistent with data from the NSABP-34 trial [218]. In premenopausal women, bisphosphonates can abrogate the bone loss associated with use of an AI. In addition, recurrence and death rates were reduced when used in combination with either tamoxifen or an AI after treatment with the LHRH agonist goserelin (ABCSG12: [219]. Taken together, these studies suggest that a bisphosphonate may have its greatest effect in a low-oestrogen environment.

The impact of bone-targeted therapy on extra-skeletal metastases and locoregional relapse also highlights the need to better understand experimental observations concerning reseeding of tumours from dormant cells within the bone microenvironment [220]. Additionally, the role of RANK-RANKL signalling in mammary stem cell biology allows for the possibility that targeting this pathway with agents such as denosumab may offer a prevention strategy for bone metastasis [221,222].

##### Oligometastatic disease

The role of localised treatment of oligometastatic disease for example in the form of selective stereotactic body radiotherapy, radiofrequency ablation or surgery is currently unclear. The impact of irradiating the primary tumour, biological communications between treated primary site and distant metastases and whether radiation therapy can convert the primary tumour into an *in situ* vaccine [223] are relatively unexplored. Prospective randomised trials are required, which should ideally incorporate comprehensive molecular studies to define subtypes most likely to respond; a related question is how to treat primary breast cancer in patients presenting with metastatic disease.

##### Radiotherapy

The molecular basis of chemo-radiosensitivity, biomarkers (including specific gene signatures, proteomic markers) of tumour and/or normal tissue sensitivity is required to allow selection of patients who may benefit from adjuvant radiotherapy and avoid toxicity to those who will not. Explanations for the mechanism(s) of favourable impacts of locoregional control from radiotherapy (RT) on survival are needed [224] and may include *in vivo* real time biosensors of tumour biology to capture transient changes in the tumour microenvironment that drive metastasis.

##### Hypofractionated adjuvant radiotherapy

Even shorter-dose fractionation schedules (that is one week of whole breast radiotherapy) might achieve equivalent locoregional control with comparable toxicity [225,226]. Partial breast irradiation appears promising, but the long-term safety and efficacy is still uncertain [197,198]. In addition, it appears likely that there is a subgroup of low-risk, older patients from whom postoperative radiotherapy can be safely omitted [227,228]. The role of postmastectomy radiotherapy in intermediate risk breast cancer [229], axillary irradiation in sentinel node positive macro- or micro-metastases [230] or boost dose in DCIS following breast-conserving surgery [231] are all currently unclear. Further definition of the role of stereotactic body radiotherapy, accounting for tumour motion [232], in combination with neoadjuvant systemic therapy, to liver or bone metastases for oligometastatic disease are required. Similarly, the optimal dose fractionation for locally advanced disease needs to be established [233].

### Molecularly targeted therapies

#### Current status

##### Anti-endocrine agents

Multiple lines of clinical and translational evidence have increased our knowledge of the risk of recurrence, particularly for ER+ve disease [212,234-236]. The optimal duration of treatment remains incompletely defined but several RCTs have provided important new data: eight to ten years of adjuvant treatment for ER+ve breast cancers is more effective than five years of letrozole or tamoxifen [237-239].

##### Endocrine therapy resistance

Comprehensive guidelines to define endocrine resistance have now been agreed [240]. Clinical studies of various agents alone and in combination with signalling inhibitors have been completed since the last gap analysis. [241-243]. The biology of ERs, including the importance of phosphorylation [244], ER co-regulators [245], cross-talk with kinases [246] and altered ER-binding events [247] nevertheless requires further elucidation. MicroRNAs regulate ER activity and endocrine responses, [248], while epigenetic events promote ER loss or tumour suppressor silencing [249]. Cancer stem cells may also be implicated in endocrine resistance [250].

The multiple cell-signalling changes driving resistance and associated disease progression, nevertheless reveal potential cancer cell vulnerabilities [251] for example mTOR [72], EGFR/HER2 [252] and Src kinase [253]. New methodologies such as large-scale siRNA screens have also provided novel therapeutic targets such as CDK10 and fibroblast growth factor receptor 1(FGFR1) [254,255].

##### Oncogenic signalling inhibitors

Several molecularly targeted therapies have been licensed since the last gap analysis including lapatinib and pertuzumab in HER2+ cancers [31] and the mTOR inhibitor everolimus in ER+ve disease [72,256], which can overcome endocrine resistance [257]. Agents targeting signal transduction pathways (notably HER2) have had a significant impact in the treatment of certain breast cancer subtypes [258]. However, there is still limited understanding of the oncogenic pathways that control the progression of premalignant breast diseases or rare, but often aggressive, breast cancers (for example metaplastic breast cancer) [259]. Molecules may have distinct functions in different cellular contexts, therefore rigorous target validation is critical [260,261]; if a signalling protein has a scaffold function, disruption of protein-protein interactions may be required for efficacy. This requires a detailed biophysical analysis of protein structures and their key interactions.

For HER-2 positive disease, dual HER-receptor blockade is more effective than monotherapy and may help prevent or overcome resistance [262,263]. Two years of adjuvant trastuzumab offers no benefit over one year [264] but the utility of shorter trastuzumab therapy is, as yet, unconfirmed [265]. In metastatic breast cancer, serum metabolomic analyses may help to select patients with HER2+ cancers with greater sensitivity to paclitaxel plus lapatinib [266]. Multiple clinical trials are evaluating PI3K pathway inhibitors; other new agents under development include HSP90 inhibitors (for example NVP-AUY922 and ganetespib); panHER, irreversible inhibitors including neratinib and afatinib; monoclonal antibodies directed against human epidermal growth factor receptor 3 (HER3) and Src inhibitors such as saracatinib.

##### Resistance to signalling inhibitors

Resistance to targeted signal transduction agents is common, arising via multiple mechanisms including utilisation of compensatory feedback loops or alternative signalling pathways. Systems biology applications have begun to describe these dynamic changes [267,268], and are critical to identify key target points for effective therapeutic intervention.

Robust guidelines (akin to REMARK) are not yet employed in studies assessing the efficacy of novel therapeutics. Such rigour is essential to ensure that both appropriate models and quantitative outputs are fully utilised. The best drug combinatorial approaches could then be developed based on mechanistic insight into opportunities afforded by synthetic lethality [269,270]. More sophisticated experimental models of DNA-damage response (DDR) defects and those that accurately reflect mechanisms of therapy resistance will enable the design of targeted therapies to overcome these clinically relevant issues.

#### What are the key gaps in our knowledge and how might they be filled?

##### Drug responses

We lack a comprehensive understanding of the exact mechanisms (both on- and off-target) by which drugs exert anti-cancer effects *in vivo*; this is exacerbated by our incomplete appreciation of networks, cross-talk and redundancy in cell signalling. Given that multiple inhibitors of specific pathways are now available (for example PI3K/PKB/mTOR), harmonised approaches to prioritisation of specific inhibitors/inhibitor classes and of research objectives in clinical trials are required.

##### Clinical determinants of intrinsic and acquired resistance

There is incomplete understanding of the role of diverse gene expression, epigenetic, protein and non-coding RNA changes in the heterogeneous manifestations of clinical resistance, [271]. There is a lack of equivalence between clinical, pathological, proliferative and molecular resistance that needs to be addressed and single genes or a canonical pathway are unlikely to be responsible. Furthermore, multiple mechanisms have also been implicated in acquired resistance, but their relationship to intrinsic resistance remains to be defined. Figure 5 illustrates the heterogeneity in patterns of gene expression in clinical endocrine resistance, suggesting that at least three major molecular mechanisms could be involved [272].

**Figure 5:** **Molecular heterogeneity of endocrine resistance.** Unsupervised hierarchical clustering of mRNA from 60 endocrine-resistant breast cancers shows heterogeneity in gene expression suggesting a multiplicity of underlying mechanisms including changes in oestrogen and interferon signalling and stromal genes. Courtesy of Professor William Miller and Dr Alexey Larionov, based on a poster presentation at the thirty-second annual CTRC-AACR San Antonio Breast Cancer Symposium, Dec 10–13, 2009 [272].

There is a need to understand the clinical impact of additional hormone receptors besides ERα, especially the progesterone receptor (PR): whilst PR is prognostic, the TEAM study has not demonstrated a predictive value [273]. Similar considerations apply to ERβ [274,275] and the androgen receptor (AR) [276], since trials of anti-androgens are currently underway in metastatic breast cancer [277].

It is not clear whether there are differences in ER+ve premenopausal vs. postmenopausal endocrine resistance [278]. As with other targeted therapies, the microenvironment, therapy-induced signalling reprogramming and stem cells are likely to play key roles. Proteomic profiling and protein functionality are particularly poorly characterised in the clinical resistance setting and such measurements remain challenging but essential.

It is important to define the contribution of CSCs to relapse on endocrine therapy, determine their sensitivity to existing agents or identify the unique signalling pathways that sustain their clonogenic potential. Diagnostic or prognostic tests based on ‘whole’ tumour samples may fail to address these potentially significant minority subpopulations of cells.

The few prospective studies to date have demonstrated that changes in management for one in six patients could be advised based on changes in breast cancer biomarkers on relapse, particularly ER, PR and HER2 [279-281]. Consequently, important clinical questions such as whether changes in the frequency of drug administration or alternating drug therapy could avoid or contribute to this process need to be addressed. Considering host factors such as adherence to medication [282], drug metabolism [283] and immune mechanisms [284], alongside molecular characteristics of tumours and the host microenvironment is essential.

##### Combinations and sequencing of targeted agents with conventional agents

Despite high-level evidence for isolated treatment situations (for example adjuvant treatment with AIs) [210,285,286], these have not been integrated into sequential treatment strategies, for example for adjuvant or first- or second-line palliative treatment. As treatment standards change (with AIs as standard adjuvant therapy), the sequence of tamoxifen as adjuvant therapy with AIs for first-line metastatic ER+ve disease may require adaptation. Such trials apply standard treatments that manufacturers may have little interest in supporting; new ways of supporting these trials will need to be explored.

Models are needed for the longitudinal study of hypoxic ‘microniches’ to inform timing of delivery of sequential targeted therapies or chemotherapy with radiation; to test real-time robotically controlled RT delivery to motion-affected hypoxic regions of primary breast tumours; and RT in combination with novel agents targeting pH regulatory mechanisms. Similarly, novel early-phase clinical trials of preoperative RT + targeted therapy or neoadjuvant hormonal therapy with baseline on-treatment biopsies for markers and gene signatures of radiosensitivity (the window of opportunity design) could complement the development of trials of stereotactic body RT to primary + neoadjuvant systemic therapy for limited-volume metastases in liver and bone.

Practical considerations include the risk/benefit of combining signalling inhibitors with anti-hormones, sequencing of tamoxifen and AIs [287] and targeting additional steroidogenic enzymes [288]. Recent randomised clinical studies have demonstrated substantial benefits for combinations of targeted agents such as endocrine therapy and mTOR inhibitors in ER+ve MBC [72] or horizontal dual HER-receptor blockade [289-292]. This results in several new challenges. Many patients benefit from single agent endocrine therapy or HER2-blockade and could avoid, at least initially, the toxicity of combination therapy if these cancers could be identified. There is a clear need to identify patients who respond adequately to targeted therapy (for example anti-HER-2 agents +/− endocrine agents) and do not need chemotherapy. Rational combinations need to be explored in the appropriate setting, taking into consideration compensatory induction of alternative signal transduction pathways bypassing targeted treatments. Treatment benefits in MBC or the neoadjuvant setting need converting into a potential survival benefit in early breast cancer.

##### New therapeutic approaches

Although phenotypically similar to BRCA1 mutant breast cancers, TNBC are heterogeneous and lack of expression of ER, PR and HER2 is not a good predictor of homologous recombination repair (HRR) status [293] Prognostic and predictive biomarkers of response for TNBC are obvious gaps which need to be addressed [294], complemented by an expanded and representative panel of fully characterised tumour cell lines and models [295]. More emphasis should be directed at developing markers of drug resistance and markers of resistance to current basal-like breast cancer/TNBC therapies [296]. Better biomarker-led characterisation could assist in patient stratification and hopefully improved treatment responses. Similarly, additional targets are required for other molecular subtypes that fail to respond to existing therapies.

##### Lymphangiogenesis and angiogenesis

Current understanding the role of lymphangiogenesis in metastasis (and thus its potential as a therapeutic target akin to neoangiogenesis) is limited [297]. In contrast, given the morbidity associated with lymphoedema following extensive lymph node dissection, identifying a means of inducing local regeneration of lymphatic vessels postoperatively could be envisaged. The contribution of the lymphatic system to immune responses to tumours is also underexplored [298]. Better *in vitro* and *in vivo* models are required to understand the cellular and molecular complexities of pathological angiogenesis and lymphangiogenesis, tumour cell intravasation, extravasation, organ colonisation and strategies for effective therapeutic interventions [299].

Anti-angiogenic therapies have been extensively trialled but have not yet lived up to their promise, with bevacizumab no longer approved for breast cancer by the FDA [300-302]. Tumour vasculature is heterogeneous [303] and multiple, temporally dynamic mechanisms contribute to the lack of durable responses [304]. The main focus has been vascular endothelial growth factor (VEGF)-driven angiogenesis but there is considerable redundancy in angiogenic signalling pathways [305]. Also, there are no validated biomarkers of response to anti-angiogenic therapies and it is likely that the vasculature of anatomically dispersed metastases will demonstrate further functional heterogeneity.

##### Exploiting the immune system

Although generally considered to be immunosuppressive, some chemotherapeutic agents (and indeed monoclonal antibodies) may involve an immune element; thus the combination of immunotherapy and chemotherapy becomes a real possibility [306,307]. In node-positive, ER-/HER2- disease, lymphocytic infiltration was associated with good prognosis in the BIG 02–98 adjuvant phase III trial [284]. There needs to be a systematic quantification of immune infiltration of breast cancer subtypes and how this relates to tumour progression, response to therapy or changes during treatment.

Cancer immunotherapy is gaining ground, whether antibody-based or cell-based, with an increasing emphasis on targeting the tumour microenvironment (for example macrophages or cancer-associated fibroblast (CAFs)) with DNA vaccines [308]. In addition, several immunogenic antigens (such as cancer testis antigens) have been detected in poor-prognosis breast cancers, which may serve as targets for therapy or chemoprevention [309,310]. New strategies for enhancing natural immunity or eliminating suppressor functions are required. There is a need for better animal models for evaluating immunotherapeutic strategies and in deciphering possible contributions to lack of responsiveness.

### Living with and managing breast cancer and its treatment

#### Current status

##### Survivorship

Cancer and its treatment have a considerable and long-term impact on everyday life [311-313]. Consequences may be physical (for example pain, fatigue, lymphoedema, hot flushes, night sweats and sexual problems), or psychological (cognitive function, anxiety, depression, fear of recurrence) and directly affect relationships, social activities and work. The relationship between the cancer patient and his/her partner will have a bearing on the level of distress: if communication is good, psychological distress will be lower [314]. Women may feel abandoned once treatment is completed with low confidence as a result [312,315]. The current system does not meet their needs [184] and the National Cancer Survivorship Initiative has been established to investigate new models of aftercare.

A recent framework publication highlights the importance of providing support to enable people to self-manage their aftercare [315]. Patients benefit from improved sense of control and ability to effect change together with an increased likelihood of seeking health information [316,317].

##### Living with advanced breast cancer

Quality of life in women with metastatic breast cancer is poor [318] with many experiencing uncontrolled symptoms [319]. Pain is a significant problem throughout the illness, not just with the end of life [318]. Depression, anxiety and traumatic stress also require intervention [320,321]. Those with metastatic breast cancer receiving social support report more satisfaction and a sense of fulfilment. Fewer avoidance-coping strategies are associated with better social functioning and a larger social network. Social stress has been found to increase pain and mood disturbance and has been associated with isolation. In addition, self-image and a decrease in sexual functioning challenge self-esteem and relationships at a time when support is most needed [322].

The impact of medical management on quality of life and decision making regarding palliative chemotherapy [323,324] and a lack of rehabilitation services [325,326] has been recognised. The convergence of palliative treatments and the end of life may impact on symptom control and care provision as well as place of death [327,328].

##### Supportive interventions

The main physical symptoms associated with breast cancer treatment are fatigue, pain, hot flushes, night sweats, cognitive and sexual problems and lymphoedema. Some interventions have demonstrated benefit with specific side effects [329-331]. Meta-analysis demonstrates that psychological interventions can reduce distress and anxiety [332], provide some physiological benefit, but with weak evidence regarding survival benefit [333]. Overall the evidence focuses on short-term benefit while the longer-term implications are unknown.

Group interventions are less effective in reducing anxiety and depression than individualised interventions such as cognitive behaviour therapy (CBT); [334], but do result in social and emotional improvements [335] and greater patient satisfaction [336]. Psycho-educational interventions show improvements in physical and psychosocial wellbeing [337] and reduced anxiety [338].

CBT reduces fatigue [339], insomnia [340] improves physical activity and quality of life [341]. CBT appears to be effective at all stages of breast cancer: group CBT can significantly reduce the impact of menopausal symptoms in breast cancer patients [342,343] with effects maintained over six months. Care packages to help improve coping skills, including group counselling sessions and/or telephone-based prompts has shown supportive care in the extended and permanent phases of survival to be effective [344]. Mindfulness-based stress reduction and cognitive therapy can improve mood, endocrine-related quality of life, and wellbeing at least in the short term [345].

Much evidence demonstrates the benefits of physical activity for breast cancer patients [346]. RCTs show that physical activity interventions during treatment show small to moderate beneficial effects on cardiovascular fitness, muscular strength and can reduce deconditioning. Post treatment, physical activity interventions result in a reduction in body fat and increase in fat-free mass, a moderate to large effect on cardiovascular and muscular strength, small to moderate effect on quality of life, fatigue, anxiety and depression and some evidence of reduced lymphoedema and osteoporosis [347,348].

The translation of physical activity research into clinical practice is a challenge. Currently, exercise-based cancer rehabilitation is not routinely incorporated into breast cancer care. However, from the National Cancer Survivorship Initiative, Macmillan Cancer Support is evaluating around 12 physical activity programmes and evaluating physical, psychological and cost benefits. One exercise intervention during therapy reassessed participants after five years and showed that those from the exercise group were still incorporating approximately 2.5 hours more physical activity a week and were more positive than control patients [349]. Furthermore, other charities are starting up similar programmes, such as Breast Cancer Care’s ‘Best Foot Forward’. There are very few intervention studies involving women with advanced metastatic cancer; these predominantly focus on supportive-expressive therapy and have been found to reduce distress [350] but the benefits are not maintained in the long term [334].

#### What are the key gaps in our knowledge and how might they be filled?

##### Inadequate translation of research findings into practice

While the problems are well recognised, there is inadequate clinical translation: for example, recognising the benefits of physical activity requires incorporating and testing intervention(s) in clinical practice. There is also a lack of representation and sensitivity to the needs of diverse groups. Similarly, the impact of breast cancer goes beyond the patient; more attention should be paid to their families, partners and children.

CBT is becoming integrated into clinical practice with training for clinical nurse specialists but there is still a need to consider how CBT and other interventions can be better integrated to widen access. Novel interventions must be developed and validated using methods based upon sound theoretical principles, with demonstrable effectiveness (both clinical and financial) that can be deployed as widely as possible to maximise benefit. A clear understanding of the components of interventions that promote uptake, adherence and long-term benefit is required. Funding for research into living with and managing the consequences of breast cancer and its treatment is very limited, adversely impacting the building of research capacity and expertise.

Establishing a multidisciplinary research consortium to develop a theoretical framework to inform research addressing the needs of those living with and managing the broad ranging consequences of breast cancer and its treatment would inform choice of outcome measures, innovative approaches to intervention design and testing. Alternative trial designs to RCTs need to be considered that incorporate patient preferences. It would also be of great benefit to the field to draw up guidance on implementing successful evidence into clinical practice.

##### Survivorship

Longitudinal studies are required to assess the recovery of health and wellbeing and the long-term adjustment of women and men who have a diagnosis of breast cancer. This will allow investigation of how unmet psychosocial needs and psychological morbidity during diagnosis and treatment relate to quality of life, sexuality, physical wellbeing and the effects of other illnesses later in life. The long-term impacts of breast cancer and therapy on everyday life need further investigation [351]. There are implications for cardiac functioning, osteoporosis, neuropathy, cognitive dysfunction, lymphoedema and shoulder mobility on the ability to maintain independence [352].

##### Living with advanced breast cancer

There is insufficient epidemiological data on the problems of women who have recurrence and metastatic disease. Research into integrated oncology and palliative care models are needed to determine which approaches improve quality of life, psychological wellbeing, palliation of symptoms, treatment decisions and end of life care. The needs of the families of women with advanced metastatic cancer and how to support them and their carers most effectively are unclear. Decision making at the end of life and the development of tools to assist women and healthcare professionals to choose appropriate treatment and place of death is needed.

##### Supportive interventions

Specialist breast care nurses have also been found to enhance the supportive care of women with metastatic breast cancer. [353]. However, there is a need to identify the active components of interventions and an individual’s preference for different types of interventions to determine what works best for him or her.

Development of mindfulness and third-wave approaches (for example Acceptance and Commitment Therapy) may be effective. More RCTs of theory-based interventions for treatment-related symptoms and innovative trial designs are needed (with longer follow-up, analysis of moderators and mediators and identified components) to support women to manage their everyday lives. Interventions to address specific psychological needs such as low self-confidence and fear of recurrence also need to be tested. Interventions are required to support women to increase their physical activity, reduce the risk of recurrence and examine the impact on late effects. The frequency, intensity, type and timing of physical activity for maximum benefit needs to be established. Effective means are required to support women to manage impaired sexuality/sexual function, altered body image, lymphoedema, weight gain [354], fear of recurrence, hormone therapy-related symptoms [341,343,355,356], cognitive problems [357][358] and post-surgical problems [359,360]. Alternative delivery of intervention needs to be explored, such as self-management, telephone or online support and non-specialist delivery: for example comparison of home-based versus hospital-based interventions on physical activity levels, patient satisfaction and motivation.

### Strategic approaches to enable progress

#### Experimental models of breast cancer

##### Improved tissue culture models

There is now a greater appreciation of the importance of employing appropriate human cancer cells. [361]. Commonly used breast cancer cell lines are derived from metastases or pleural effusions and fail to adequately represent the diversity and complexity of breast cancer [362]. It has proven difficult to establish human tumour cell cultures representative of the major subtypes and to maintain their genomic and phenotypic integrity. In addition, inter-patient variability and inadvertent selection of the most malignant subtypes, skews availability of representative material.

Better representation of breast cancer subtypes is required. Material from normal mammary tissue, premalignant breast conditions, different ER+ve (and rare) subtypes of breast cancers and ideally metastases from all major sites are needed to cover the full spectrum of breast cancer development and progression. Primary or minimally passaged cell cultures will avoid issues of misidentification, contamination or long-term culture artefacts. Ideally, a central repository of well-annotated human primary breast cancer cells, associated host cells and cell lines should be available to researchers linked to a searchable, open-access database. Maintaining breast tumour tissue in culture with its essential characteristics intact will enable prognostic screening and testing of potential therapeutic agents.

Reliable cell-type-specific markers are required and it is also important to be able to recognise cancer stem cell subpopulations (or transient phenotypes). Identification of promoters for distinct cell subpopulations will enhance the number and scope of available *in vitro* models. [363] and enable conditional genetic modifications for mechanistic and target validation studies [364]. Ideally, co-cultures (of both normal and precancerous breast cells) with host cell populations such as fibroblasts, myoepithelial cells, macrophages, adipocytes or vascular endothelial cells are needed for studies of cellular interactions within the appropriate ECM microenvironment.

Three-dimensional culture models can recapitulate the tissue architecture of the breast and its characteristic invasion patterns [89,365] especially if host stromal components are incorporated [366]. Three-dimensional heterotypic model systems are also enabling dissection of the effect of cell-cell interactions and stromal elements in drug resistance. Three-dimensional cultures require additional refinement, higher throughput, quantitative assays [367] and a move towards more physiologically relevant conditions, for example by the use of bioreactors, enabling long-term cultures under flow conditions; especially appropriate for invasion assays [368,369].

##### Animal tumour models

In the last five years there has been an expansion in the use of orthotopic (anatomically correct) breast cancer xenografts [370] and significant advances in developing patient-derived xenografts (PDX) [371]. These models better reflect the human cancers from which they were derived and ER+ve tumours respond appropriately to oestrogen ablation [372]. Increased use of genetically engineered mouse (GEM) models driven by relevant abnormalities such as BRCA mutations, HER2 overexpression and so on have enabled the study of naturally occurring tumours in immunocompetent hosts and evaluation of new targeted therapies such as PARP inhibitors and the emergence of resistance [373]. Pros and cons of different models are shown in Figure 6.

**Figure 6:** **Comparative properties of experimental tumour models.***In vitro* assays of tumour growth and response to therapy can be conducted in two dimensions or three dimensions - the latter more closely approximating the biology of solid tumours than a simple monolayer. Cultures can be enhanced by the addition of matrix proteins and/or host cells and can be adapted to measure not only tumour cell proliferation, but also additional cancer hallmarks such as invasion. Standard *in vivo* assays depend upon the transplantation of established human tumour cell lines into athymic (immune-incompetent) hosts. These models are relatively simple and easy to use, but are increasingly complemented by genetically engineered mice harbouring targeted genetic mutations which render them susceptible to developing mammary cancers. The figure summarises key advantages and disadvantages of each model and means by which their clinical relevance and utility might be enhanced. Based on a figure provided courtesy of Claire Nash in Dr Valerie Speirs’ group (University of Leeds).

Expansion of PDX models will be required to cover all the main breast cancer phenotypes [374] and to address the contribution of ethnic diversity [375]. Advanced GEM models with multiple genetic abnormalities, able to generate both hormone sensitive and insensitive tumours and in which metastasis occurs at clinically relevant sites will also be a desirable refinement [376,377]. However, all such animal models will require validation of any findings in the clinical setting [296,378,379]. Models are also required to investigate mechanisms of the induction of (and escape from) long-term tumour dormancy [380], a unique feature of breast cancer.

Invasive behaviour does not occur uniformly or synchronously within a tumour [381] and this heterogeneity is not easily reproduced *in vitro*. Improved tumour models and methods are required to understand the localised and possibly transient factors involved in temporal and spatial heterogeneity that promote invasion and metastasis.

##### Models for testing novel targeted agents against disseminated disease

Novel agents designed for systemic administration are rarely tested against established invasive/metastatic disease in preclinical animal models [382,383]. There is an urgent need to develop better models for the discovery and development of therapies targeting metastases that are effective against all sites of disease [384].

In around 20% of women, complete resection of primary tumours does not prevent distant metastases because dissemination has already occurred. In these cases, agents targeting cell motility or invasion may have limited value. It is therefore critical that preclinical models used for testing such therapies incorporate established micrometastases [385]. Similarly, there is a preponderance of lung metastasis models in routine use. Other important sites of breast cancer metastasis (for example bone, brain and, liver) are relatively poorly represented, and this needs remedying in preclinical drug evaluation [386-388]. Human tissue (such as bone) transplanted into mice can provide a more relevant microenvironment [389].

Preclinical or clinical trials focused on tumour shrinkage are not appropriate for testing the efficacy of anti-invasive or anti-metastatic agents that may reduce metastasis without significantly impacting primary tumour growth [390]. Such approaches would likely fail current response evaluation criteria in solid tumors (RECIST) criteria and show little activity in the neoadjuvant setting or in late stage patients with advanced metastatic disease. The potential to utilise veterinary models for testing novel therapies or RT-systemic therapy combinations and cross-disciplinary collaboration with other scientific disciplines to develop real-time *in vivo* biosensors of tumour biology offer novel opportunities for significant progress.

##### Modelling drug resistance

While challenging, establishing cell lines, tissue slice models and PDX from relapsed and resistant cancers should be the ultimate goal in order to provide a window on the mechanisms that occur in patients where therapies fail. This would also allow *ex vivo* targeting studies, employing signalling analyses and imaging systems to track resistance mechanisms and progression.

Preclinical endocrine resistant models have largely been derived from ER+ve MCF7 cells *in vitro*, either by transfection of potential signalling molecules such as HER2 or from continuous exposure to anti-endocrine agents. Extensive panels of relapsed human tumour cell lines are required to reflect the heterogeneity of clinical resistant disease. This will allow assessment of the impact of genetic background, duration, sequence and type of endocrine agent (including AI) and rational evaluation of agents to reverse resistance [391]. It is critical to validate mechanisms identified *in vitro* with clinical resistance.

##### Longitudinal clinical samples and associated biological studies

Biobanking has substantially improved and is seen as a significant outcome of the last gap analysis [7] but the systematic analysis of clinical material collected from serial tumour biopsies/ fine-needle aspiration (FNA) (or ideally less invasive means such as ‘liquid biopsy’) before, during and following resistance development is lacking. Procurement of matched materials remains challenging but is critical to establishing clinically relevant signalling mechanisms that culminate in acquired resistance, allowing tracking of the dynamics and prevalence of molecular events during response through to any subsequent relapse. Care must be taken to provide adequate sampling of inherently heterogeneous tumours in their primary, recurrent and disseminated settings, which may also provide material for study of site-specific metastasis. [392] and samples must be full annotated, ideally with ‘omics’ profiling and immunohistochemistry. The biopsy of metastatic lesions is challenging and will require systematic introduction of a ‘warm autopsy’ programme [393]. A more realistic alternative is to further exploit the preoperative neoadjuvant setting, despite the potential issues of heterogeneity and sampling [394]. Collection of such samples is a particularly valuable resource to address mechanisms of intrinsic resistance and to track early therapy-associated signalling changes (Figure 7).

**Figure 7:** **Longitudinal sampling and enhanced biobanks.** The longitudinal collection of blood and samples from normal breasts, primary cancers and relapsed/metastatic/treatment-resistant disease is essential in order to address the origins, heterogeneity and evolution of breast cancers. Samples are required from as broad a patient population as possible to understand ethnic, age-related and gender differences in incidence, molecular subtypes, prognosis and response to treatment. Sequential samples (ideally patient-matched) from primary tumours and metastases will enable detailed studies of tumour evolution/progression and provide material for generating new cell lines and patient-derived xenografts for translational research. Multimodality imaging and metabolomic analyses will add further dimensions of valuable information. Based on a figure provided courtesy of Professor William Gallagher, with thanks to Dr Rut Klinger (UCD Conway Institute).

Increased use of clinical relapse material will determine the relevance of preclinical findings and identify potential candidates for detailed mechanistic evaluation in appropriate tumour model systems. Ultimately the goal is to determine if patients can be better stratified to allow rational, personalised choices for further therapy. This aspiration requires better integration between clinicians and scientists, trial providers and pharmaceutical companies and would benefit from data sharing. Tissue-based analyses from clinical trials need to be expanded to incorporate all of the next generation sequencing studies for research. These initiatives need to be co-ordinated with cancer registry/ British Association of Surgical Oncology (BASO) breast cancer data.

Blood samples for early diagnosis, monitoring treatment response, early indicators of disease relapse (and revealing increased heterogeneity) are imperative as our ability to generate new biomarkers through emerging technologies increases. These include detection of CTCs, miRNAs, ctDNA, exosomes, and so on. Serum HER2 measurement may be another promising biomarker with prognostic and predictive value [395-398].

##### Biomarkers of response or relapse

With the exception of ER and HER2, the availability of biomarkers to accurately identify which patients will receive benefit from targeted treatment, and indicators of patients at high risk of progression or relapse remains limited. Further advances in molecularly targeted and anti-endocrine therapy require clinically applicable predictive biomarkers to enable appropriate patient recruitment and to track responses to treatment [399,400]. These analyses should be applied both to primary tumours and recurrent/metastatic lesions to accommodate the profound heterogeneity within individual cancers, which increases further during disease progression. Understanding which molecular markers are ‘drivers’ of breast cancer and their functional roles at different stages of disease will be key to designing more effective targeted agents.

Validation of predictive markers for drug response could be better facilitated by the routine inclusion of such approaches into clinical trials rather than retrospective analyses of archived material. Any new biomarkers should have well-defined cut-off points, be thoroughly validated and robust. We require biomarkers to identify patients who will *not* respond to trastuzumab (primary resistance) in addition to the development of secondary acquired resistance. Discriminatory biomarkers are required for combination therapies such as lapatinib and trastuzumab in HER2-positive breast cancers. We lack preclinical data that can predict which combination of anti-HER2 therapies is optimal. There is also a need for biomarkers that can identify patients who may be more suitably treated with a tyrosine kinase inhibitor (TKI) rather than trastuzumab or combination anti-HER2 therapy. New irreversible TKIs currently in clinical trials, (for example afatinib and neratinib) have shown increased potency in preclinical studies - could these now become the mainstay for HER2-positive tumours?

Knowledge of the therapeutic benefits of mTOR inhibitors and of newer PI3K pathway inhibitors in breast cancer subtypes is rudimentary and we have no biomarkers that can be used to optimise their therapeutic index. In addition, knowledge of how important genomic (for example *PIK3CA* mutations) and proteomic (for example PTEN loss) biomarkers impact the efficacy of specific PI3K pathway inhibitors in the clinical setting is limited. Further preclinical research on the functional proteomic effects of genomic abnormalities in the PI3K pathway in breast cancer is essential.

ER+ve tumour heterogeneity remains a challenge: luminal A vs. luminal B subgroups impact on prognosis; however, the mechanisms of endocrine failure remain largely unknown. In ER+ve disease there is a lack of accepted biomarkers/signatures to distinguish endocrine-sensitive patients from those with intrinsic insensitivity or who will develop early or late resistance.

There is a need to develop non-invasive means of detecting risk of subsequent relapse. In addition to serial tumour samples, serum samples are warranted as these may ultimately provide less invasive indicators of acquisition of resistance. It remains unclear if single or multiple biomarkers or transcriptional profiles are optimal, or even if basic endocrinological markers may prove valuable in the context of predicting resistance.

##### Imaging

While imaging (at least with some modalities) is routinely applied to the early detection and follow-up of breast cancers, there is a need to increase the use of functional screening techniques to better understand tumour heterogeneity, identify features associated with response or resistance to treatment and more rapidly translate promising new preclinical methodologies to clinical evaluation. It is important to evaluate emerging imaging biomarkers of primary and metastatic breast cancer and there is a requirement for new, more specific and clinically translatable radiotracers for positron emission tomography/single-photon emission computed tomography (PET/SPECT) [401,402]. We also need to identify and assess the utility of imaging biomarkers associated with other hallmarks of cancer beyond proliferation for example invasion, altered metabolism, hypoxia. Attention needs to be given as to how to validate novel imaging biomarkers in adequately powered multi-centre clinical trials. The funding available from most grant-awarding bodies is insufficient to cover this, suggesting the need to consider larger collaborative trials funded by more than one agency.

Imaging may also be able to report on intratumoural heterogeneity and identify the most significant region (for example more aggressive/invasive areas via diffusion-weighted magnetic resonance imaging (MRI)), to more accurately direct biopsies or radiotherapy. EMT could be addressed by the increased use of cluster, histogram and/or texture analyses, but it will be necessary to define the correct metrics to assess and quantify such phenotypes [403]. It would be desirable to extend these techniques to define different tumour subtypes such as DCIS, luminal or TNBC non-invasively (which may identify mixed lesions missed by homogenised or limited sample analyses) and assess heterogeneity between metastases. Ideally, imaging studies (both preclinical and clinical) should be co-registered with linked genomic and proteomic information in order to fully interpret the biological relevance of the images obtained [404-406]. However, tissue collection is often not co-ordinated with imaging studies and the added benefit not always appreciated.

A key achievable goal is to non-invasively evaluate predictive biomarkers of therapeutic responses. Increased adoption of more clinically relevant orthotopic xenograft and transgenic murine models of primary and metastatic breast cancer will demand robust preclinical imaging approaches. The use of such models in imaging-embedded trials of novel agents will improve the accuracy of preclinical data, accelerating the development of promising drugs, or enabling early closure of suboptimal programmes. Such refined preclinical trial designs will also prove highly informative in establishing combination and/or sequential treatment regimes.

##### Clinical trial design and patient involvement

Clinical trial design should be adapted to use preoperative and neoadjuvant models to allow novel therapies to be tested in patients [394,407], identify *de novo* resistant cancers and investigate how such resistance can be counteracted. These approaches are particularly relevant for therapeutic strategies that target cancer stem cells, residual (dormant) cancer cells or influence the tumour microenvironment. Future trial design will also have to incorporate dynamic strategies, such as using the response to short-term treatment to guide the use of additional preoperative treatment. Given the increasing focus on small target populations (for example molecular subtypes of breast cancer), clinical trial strategies for effective patient stratification or selection based on molecular characteristics are required to allow routine integration into large-scale clinical trials. In addition, the relatively long period between surgery and relapse in breast cancer patients impacts negatively on the economic feasibility of such clinical trials. New thinking will be required to modify clinical trial design, and to consider biomarkers that relate to invasive and metastatic phenotypes, for example as in trials with denosumab where the development of skeletal-related events (SRE) was an accepted and measurable endpoint [221].

##### Patient reported outcomes

There is a need to incorporate standardised patient-reported outcome measures (PROMs) both within clinical trials and in everyday clinical practice. Currently, many trial reports are reliant on the common terminology criteria for adverse events (CTCAE) gradings about side effects, which show alarming discrepancies with data actually collected from patients [408].

##### Psychosocial considerations

Further research is needed to support the use of decision aids around surgery and treatment and to define any benefits. There is also a need for prospective research to identify consequences of treatment and the impact of co-morbidities on the lives of women with breast cancer so that future patients can consider these as part of their decision making. The experiences of minority ethnic groups, younger (<45 years) and older (>70 years) women in relation to their treatment choices and management need further research. Addressing non-adherence to endocrine therapy and understanding the biological mechanisms of significant side effects such as menopausal symptoms are poorly understood. The value of incorporating lifestyle recommendations as part of routine care and its impact on recovery and quality of life should be further explored.

##### Multidisciplinary collaborations and resources

Increased resources are required to support core (for example biochemical/IHC) as well as new ‘omics technologies; to develop improved *in vitro*/*in vivo*/*ex vivo* model development, serial clinical sample collection, advanced bioinformatic/systems biology analysis, clinical biomarker validation and ‘bench to bedside’ drug development. Stronger multidisciplinary collaborations between laboratory scientists, clinicians, bioinformaticians and engineers (and in turn with funding bodies and industry) must be encouraged. Much better integration of computer science, database engineering, data analytics and visualisation, hardware and software engineering within biological research will be essential to effectively read and translate increasingly complex data. Convincing drug companies of the benefits of a co-ordinated approach (tissue collection before, during and after treatments) in clinical trials of new drugs is problematic, and access of material for research purposes is limited. Companies must be convinced of the benefits of accurate biomarkers to allow for the better stratification of patients. Even though this will limit their target population, this should be offset by higher response rates and faster regulatory approval.

Continued support is required for basic biological research and understanding of cell signalling processes with emphasis on interactions, cross-talk and microenvironmental regulation. It is important that approaches in this area are linked to systematic investigations and precise analyses of cell responses to a wide range (and combination) of inhibitors, tested in clinically relevant breast cancer model systems. A key element is open discussion and learning from negative results to avoid unnecessary duplication of research. Sharing of information, best practice, optimised model systems, technologies and resources is essential, perhaps through developing web-based analysis portals. Such approaches are needed to integrate and interpret diverse sources of data to understand the plasticity of signalling emerging during treatment though to resistance (Figure 8).

**Figure 8:** **Integrated vision of multidisciplinary research.** Enhanced integration and utilisation of the vast amount of clinical and experimental observations relating to breast cancer is urgently required. Clinical observations generate hypotheses relating to the origins of cancer, its underlying molecular pathology and potential vulnerabilities that could be exploited for therapeutic benefit. Such insights provide opportunities for testing and validation in *in vitro, in vivo* and *in silico* models. Drug discovery aims to provide inhibitors of major oncogenic ‘drivers’ for use singly or in combination with conventional therapies; such personalised medicine requires the co-development of predictive and pharmacodynamic biomarkers of response. Results from preclinical therapy studies and clinical trials should be fed back into searchable databases to reveal reasons for treatment failure and allow new strategies to be tested and deployed. Based on a figure provided courtesy of Professor William Gallagher, with thanks to Professor Walter Kolch (UCD Conway Institute).

A co-operative network of advanced radiotherapy facilities, analogous to the Experimental Cancer Medicine Centres is needed to ensure adequate patient numbers for clinical trials. Engaging patients and healthcare teams is critical to enable complex biological studies (especially longitudinal biomarker studies). Lack of academic clinicians (particularly in radiation oncology), radiobiology and physics staff nationally and rising service pressures on NHS staff are all detrimental to delivery of clinical translational research.

## Conclusions

While substantial advances have been made in breast cancer research and treatment in the last five years, there remain significant gaps in translating this newly acquired knowledge into clinical improvements.

Understanding the specific functions and contextual interactions of genetic and epigenetic advances and applying this knowledge to clinical practice, including tailored screening, will require deeper understanding of molecular mechanisms and prospective clinical validation. Even with clinically actionable tests, decision making, support for patients and their families and overcoming the barriers to lifestyle change (diet, exercise and weight) alongside chemopreventive strategies are required to optimise health outcomes.

Genomic profiling of sequential clinical samples (primary, relapsed and secondary cancers, CTC, ctDNA, before, during and following therapy) is required to identify specific biomarkers of inter-/intra-tumour spatial and temporal heterogeneity, metastatic potential, sensitivity to radiotherapy and different forms of chemotherapy, *de novo* or acquired resistance. This will significantly improve patient stratification for existing therapies and identify key nodes in these dynamic processes as potential new therapeutic targets. Validated markers of these processes (including minimally invasive multimodality imaging and metabolomics methodologies) will benefit from synergies between laboratory and clinical interactions. Improved understanding of the interactions, duration, sequencing and optimal combinations of therapy should allow better stratification of patients and reduce overtreatment (or undertreatment) enhancing prevention or survival while reducing morbidity.

Further genetic, epigenetic and molecular profiling of breast cancers and their associated stroma would be significantly enhanced by expanded panels of cell lines representing all major breast cancer subtypes and three-dimensional tumour-host heterotypic co-culture systems. This would enable increased understanding of the molecular drivers behind specific cancer subtypes and their role (together with microenvironmental modifiers) in treatment resistance and metastasis. Deciphering tumour-stromal interactions incorporating metabolic and immunological host mechanisms and intracellular/extracellular signalling pathways would have therapeutic implications for prevention and therapy. Advanced high-content analytical methods will enable consideration of additional key cancer ‘hallmarks’ beyond proliferation (for example cell motility and invasion) and enable screening for inhibitors under more physiologically relevant conditions. Better preclinical animal models (for example genetically engineered mice expressing relevant human oncogenes, which develop widespread metastases; patient-derived xenografts) are required. Such models would enable testing of hypotheses derived from clinical observations and rigorous target validation and evaluation of novel therapies in the metastatic setting (and where desirable in immunocompetent hosts).

Underpinning these advances, optimised multimodality imaging for diagnosis and therapeutic monitoring should enable better evaluation of primary and metastatic disease. Clinically annotated tissues for translational research must be linked to bioinformatics as key contributors to interdisciplinary research, essential for rapid future advances. Increasing numbers of women and men are surviving breast cancer. Alongside advances in understanding the disease and using that knowledge for prevention, earlier detection and successful treatment of breast cancer, interventions to improve the survivorship experience require innovative approaches to address the consequences of diagnosis and treatment.

Top 10 gaps:

1. Understanding the specific functions and contextual interactions of genetic and epigenetic changes in the normal breast and the development of cancer

2. Effective and sustainable lifestyle changes (diet, exercise and weight) alongside chemopreventive strategies

3. Tailored screening approaches including clinically actionable tests

4. Molecular drivers behind breast cancer subtypes, treatment resistance and metastasis

5. Mechanisms of tumour heterogeneity, tumour dormancy, *de novo* or acquired resistance; how to target the key nodes in these dynamic processes

6. Validated markers of chemosensitivity and radiosensitivity

7. Interactions, duration, sequencing and optimal combinations of therapy for improved individualisation of treatment

8. Optimised multimodality imaging for diagnosis and therapeutic monitoring should enable better evaluation of primary and metastatic disease

9. Interventions and support to improve the survivorship experience including physical symptoms such as hot flushes and lymphoedema

10. Clinically annotated tissues for translational research including tumour, non-tumour and blood based materials from primary cancers, relapsed and metastatic disease

Proposed strategic solutions:

For significant progress to be made in treating and supporting those impacted by breast cancer (and ultimately preventing and overcoming this disease) basic and translational research scientists in academia and industry, funding bodies, government and patients need to work together to achieve the following key strategic solutions

1. To reverse the decline in resources targeted towards breast cancer research, funding must be increased and strategically directed to enhance our current knowledge, develop the talent pool, and apply evidence-based findings to improve clinical care

2. A fully cohesive and collaborative infrastructure must be developed to support breast cancer research; this requires improved access to appropriate, well-annotated clinical material including longitudinal sample collection with expert bioinformatics support and data sharing.

3. Building on sound investment and infrastructure, all stakeholders (researchers, funders, government, industry and patients) must work together on the clinical development and translation of research knowledge to patient benefit. For example, enhanced, clinically relevant, *in vitro* and *in vivo* models are required for evaluation of new therapies together with validated biomarkers, which should then be embedded in clinical practice.

4. Research funders, government and industry should provide innovative programmes to encourage collaborative cross-disciplinary working practices, including the training of more physician-scientists and integration of physical sciences, technology and engineering.

5. Improving clinical trial methodologies, including patient involvement, recognising that a changing global environment is required to ensure that all clinical developments can be tested and ultimately implemented for patient benefit.

## Abbreviations

AI: Aromatase inhibitor; AR: Androgen receptor; ATM: Ataxia telangiectasia mutated; BASO: British Association of Surgical Oncology; CAF: Cancer-associated fibroblast; CBT: Cognitive behavioural therapy; CDK10: Cyclin-dependent kinase 10; CHEK2: CHK2 checkpoint homolog; CHK2: Checkpoint kinase 2; CNS: Central nervous system; CSC: Cancer stem cell; CTC: Circulating tumour cell (in blood); CTCAE: Common terminology criteria for adverse events; ctDNA: Circulating tumour DNA; DCIS: Ductal carcinoma *in situ*; DDR: DNA damage response; DNA: Deoxyribonucleic acid; DTC: Disseminated tumour cell (usually in marrow nodes or tissue); ECM: Extracellular matrix; EMT: Epithelial-mesenchymal transition; ER: Oestrogen receptor; FGF: Fibroblast growth factor; FGFR1: Fibroblast growth factor receptor 1; FNA: Fine-needle aspiration; FOXA1: Forkhead box protein A1; GEM: Genetically engineered mouse; GWAS: Genome-wide association studies; HER2: Human epidermal growth factor receptor 2; HER3: Human epidermal growth factor receptor 3; HRR: Homologous recombination repair; HRT: Hormone replacement therapy; HSP90: Heat shock protein 90; IBTR: Ipsilateral breast tumour recurrence; ICGC: International Cancer Genome Consortium; ICOGs: Illumina collaborative oncological gene-environment study; IGF1: Insulin-like growth factor 1; IHC: Immunohistochemical; iPS: Induced pluripotent stem cells; LC-MS: Chromatography-mass spectrometry; MBC: Metastatic breast cancer; miRNA: Micro RNA; MRI: Magnetic resonance imaging; NMR: Nuclear magnetic resonance; panHER: Representing the whole HER family; PARP: Poly (ADP-ribose) polymerase; PDX: Patient-derived xenografts; PET/SPECT: Positron emission tomography/single-photon emission computed tomography; PI3K: Phosphatidylinositide-3 kinase; PIK3CA: Gene encoding PI3 kinase alpha; PKB: Protein kinase B; PR: Progesterone receptor; PROMs: Patient-reported outcome measures; RCT: Randomised controlled trial; RECIST: Response evaluation criteria in solid tumors; RNA: Ribonucleic acid; RT: Radiotherapy; SERMs: Selective oestrogen receptor modulators; siRNA: Short inhibitory RNAs; SNB: Sentinel node biopsy; SNP: Single nucleotide polymorphism; SRE: Skeletal-related events; START A: Standardisation of Breast Radiotherapy (START) trial A; START B: Standardisation of Breast Radiotherapy (START) trial B; TCGA: The Cancer Genome Atlas; TGFβ: Transforming growth factor beta; TKI: Tyrosine kinase inhibitor; TMA: Tissue microarray; TNBC: Triple-negative breast cancer; VEGF: Vascular endothelial growth factor; WHI: Women’s Health Initiative.

## Competing interests

Dr Galina Velikova: Chair of a working group of the National Cancer Survivorship Initiative led by Macmillan Cancer Support.

Drs Helen Bryant and Dr Nicola Curtin: hold patents for PARP inhibitors.

Professor William Gallagher: co-Founder and part-time Chief Scientific Officer of OncoMark, a molecular diagnostics company.

Dr Martin Leach: director of Specialty Scanners plc, developing MRI-based diagnosis and treatment systems.

Dr Sacha Howell: Advisory Board honoraria from AstraZeneca, Roche, Novartis, Genomic Health and Celgene.

Dr Robert Stein: shareholder in GlaxoSmithKline and chief investigator of the OPTIMA study; travel funds received from Celgene, Roche, BristolMeyersSquibb, SanofiAventis and Novartis; Advisory Board fees from Novartis, Amgen, GSK, Roche and AstraZeneca.

Dr Nigel Bundred has received paid honoraria from Genomic Health.

The remaining authors declare that they have no competing interests.

## Authors’ contributions

*denotes recipient of Breast Cancer Campaign funding in the last five years. ^≠^ denotes current Breast Cancer Campaign Scientific Advisory Board membership. ^#^ denotes current Breast Cancer Campaign Board of Trustees membership. Chairs: SAE^#^ and AMT^#^ conceived the overall strategy, designed the workshop formats and authored the manuscript on the basis of the final reports submitted by the nine working groups. Group Leaders: RBC, IDSS, DGE*^≠^, CF^≠^,WMG^≠^, AH^≠^, IH*^≠^, LJJ*, SPL, SPR^≠^, PS*^≠^, and VS* led their respective groups with the help of the Deputy Group Leaders, co-ordinated responses from a pre-circulated questionnaire, and wrote and submitted final reports. Deputy Group Leaders: EOA, NJB ^a^, JMF*^≠^, JMWG*, AJH*, MH, AK, JRM*, PM*^≠^, ES, MJS*^≠^, ER, and RN* supported the activities of the Group Leaders in contributing to collating workshop presentations and discussions and producing the final reports from each group. Working group members: SA*, ASA , JA*, FB*, JPB*, KB*^≠^, NJB^b^, HEB^≠^, JMB, AMC*, JSC*, CEC*, GJRC*, AC, NJC, LVD*^≠^, SWD, DFE, DME, DRE*, JE, DFF*, MGC, AJG, VG, AMG, BTH, SH, SJH^≠^, GH, NHW, MSH, BJ, TJK, CCK, IHK*, MOL, DJM, JFM*^≠^, LAM, SGM^≠^, JEM, DWM, WRM, JRM, SMM*, JPBOC, ROC*, CP, PDPP*, EAR^≠^, JMS*, RS^≠^, JS, CHS, ANJT, GV, RAW*, CJW, KJW^≠^ and LSY all participated in/contributed to the gap analysis workshops, discussions and in generating the respective reports. NJB^a^ Nigel J Bundred. NJB^b^ Nicola J Brown. All authors read and approved the final manuscript.
